RETRACTED

# Analysis and Validation of Differentially Expressed Ferroptosis-Related Genes in Regorafenib-Induced Cardiotoxicity

**DOI:** 10.1155/2022/2513263

**Published:** 2022-09-26

**Authors:** Siyuan Zhang, Xueming Xu, Zhangyi Li, Tian Yi, Jingyu Ma, Yan Zhang, Yilan Li

**Affiliations:** ^1^The Second Affiliated Hospital of Harbin Medical University, Harbin, Heilongjiang 150000, China; ^2^Department of Biochemistry and Life Sciences, Faculty of Arts and Sciences, Queen's University, Kingston, Ontario, Canada 91761; ^3^Harbin Medical University, Harbin, Heilongjiang 150000, China; ^4^Key Laboratory of Myocardial Ischemia, Ministry of Education, Harbin Medical University, Harbin, Heilongjiang 150000, China

## Abstract

**Background:**

Although tyrosine kinase inhibitors (TKIs) constitute a type of anticancer drugs, the underlying mechanisms of TKI-associated cardiotoxicity remain largely unknown. Ferroptosis is a regulated cell death form that implicated in several tumors' biological processes. Our objective was to probe into the differential expression of ferroptosis-related genes in regorafenib-induced cardiotoxicity through multiple bioinformatics analysis and validation.

**Methods and Materials:**

Four adult human cardiomyocyte cell lines treated with regorafenib were profiled using Gene Expression Omnibus (GEO) (GSE146096). Differentially expressed genes (DEGs) were identified using DESeq2 in *R* (V.3.6.3). Then, Gene Ontology (GO) Enrichment Analysis, Kyoto Encyclopedia of Genes and Genomes (KEGG) Enrichment Analysis, and Gene Set Enrichment Analysis (GSEA) were used to explore DEGs' bioinformatics functions and enriched pathways. We intersected DEGs with 259 ferroptosis-related genes from the FerrDb database. Finally, the mRNA levels of differentially expressed ferroptosis-related genes (DEFRGs) were validated in regorafenib-cultured cardiomyocytes to anticipate the link between DEFRGs and cardiotoxicity.

**Results:**

747,1127,773 and 969 DEGs were screened out in adult human cardiomyocyte lines A, B, D, and E, respectively. The mechanism by which REG promotes cardiotoxicity associated with ferroptosis may be regulated by PI3K-Akt, TGF-beta, and MAPK. GSEA demonstrated that REG can promote cardiotoxicity by suppressing genes and pathways encoding extracellular matrix and related proteins, oxidative phosphorylation, or ATF-2 transcription factor network. After overlapping DEGs with ferroptosis-related genes, we got seven DEFRGs and found that ATF3, MT1G, and PLIN2 were upregulated and DDIT4 was downregulated. The ROC curve demonstrated that these genes predict regorafenib-induced cardiotoxicity well.

**Conclusion:**

We identified four DEFRGs which may become potential predictors and participate in the regorafenib-induced cardiotoxicity. Our findings provide possibility that targeting these ferroptosis-related genes may be an alternative for clinical prevention and therapy of regorafenib-related cardiotoxicity.

RETRACTED

## 1. Introduction

The burden of cancer incidence and mortality are increasing rapidly around the world according to GLOBOCAN, a global cancer statistics program conducted by the International Agency for Research on Cancer [1]. In the past few decades, anticancer treatment has achieved remarkable success, dramatically improving the outcomes of cancer patients. However, the side effects brought by these anticancer therapies cannot be underestimated. Cardiotoxicity is typically defined as toxicity that adversely affects the heart and may eventually lead to cardiomyopathy [2]. A variety of anticancer drugs, such as immune checkpoint inhibitors (ICIs), TKIs [3], proteasome inhibitors [4], and microtubule inhibitors [5], have shown to exert harmful effects on the cardiovascular system through their own toxic effects or increasing the side effects of other drugs [6]. Moreover, some of them [7] could induce life-threatening cardiotoxicity such as ischemia, infarction, arrhythmia, and damage to cardiac valves, the conduction system, or the pericardium [8]. Given the extensive application of novel anticancer therapeutics, exploring potential mechanisms, finding reliable prediction biomarkers, and providing possible treatment targets of anticancer drug-induced cardiotoxicity are of particular importance.

Regorafenib (REG) is an FDA-approved small molecule TKI utilized in treating patients with colorectal cancer (CRC), gastrointestinal stromal tumors (GIST), and hepatocellular carcinoma (HCC) [9]. Given that REG exhibit multitarget pharmacology, inhibition of multiple protein kinases in cardiomyocytes may also lead to adverse cardiovascular events such as hypertension, myocardial ischemia, and infarction [10]. A meta-analysis showed that in 6 randomized, placebo-controlled clinical trials of 2065 patients, the REG treatment group significantly increased the risk of hypertension and hemorrhage compared with the control group [11]. In addition, cellular mitochondrial membrane potential and mitochondrial complex I and V protein levels were reduced in cardiac cells treated with high doses of REG (20 mM), suggesting that REG-induced cardiotoxicity may be related to mitochondrial damage [12]. Nonetheless, there is very relatively little information available about the precise molecular mechanisms underlining REG-induced cardiotoxicity.

Ferroptosis is a new iron-dependent cellular death mechanism produced by lipid peroxidation following suppression of the cystine/glutamate antiporter system, leading to the rupture of plasma membrane [13]. According to previous studies, ferroptosis is attributed to multiple disorders, particularly tumors, cardiovascular diseases, and neurodegenerative diseases [14–16]. Iron overload can lead to decreased viability of bone marrow mesenchymal stem cells [17]. Gao et al. demonstrated that mitochondria played a crucial part in ferroptosis caused by cysteine deficiency, contributing to tumor suppression [18]. Additionally, it is noteworthy that mitochondrial-dependent ferroptosis also participated in doxorubicin-induced cardiotoxicity [19]. Moreover, cotreatment of human ovarian cancer cells with PACMA31- and REG-induced ferroptosis could be fully blocked by ferrostatin-1 [20]. However, whether ferroptosis participates in REG-induced cardiotoxicity, which ferroptosis-related genes are involved and how these molecules contribute to cardiotoxicity, remains largely unknown.

RETRACTED

In this study, the purpose is to explore the connection between ferroptosis and REG-induced cardiotoxicity using multiple bioinformatics methods and experimental validation. The differentially expressed ferroptosis-related genes (DEFRGs) identified by our study may function as the ferroptosis-related biomarkers for disease diagnosis and therapeutic monitoring.

## 2. Materials and Methods

### 2.1. Acquisition of Data and Study Design

Supporting the present study, we screened and obtained mRNA expression datasets (GSE146096) for transcriptomic profiling of four adult human heart-derived primary cardiomyocyte lines treated with REG from the GEO database (https://www.ncbi.nlm.nih.gov/GEO/). Then, the four groups of human heart-derived primary cardiomyocytes treated at the same REG concentration and the same treatment time (concentration: 1 nM; treatment time: 48 hrs) were divided into lines A, B, D, and E, respectively. There were 6 control groups and 2 REG treatment groups in A line, 9 control groups and 3 REG treatment groups in B line, 6 control groups and 3 REG treatment groups in D line, and 11 control groups and 4 REG treatment groups in E line. The data collecting and analysis process is presented in Figure 1.

The FerrDb database (http://zhounan.org/ferrdb) was used to download 259 ferroptosis-related genes, which comprised of drivers, suppressors, and markers of ferroptosis.

### 2.2. Differential Gene Expression

The control and REG treatment groups of the four transcriptomic profiling groups were compared separately, and statistical analysis and visualization were performed using the DESeq2 package in the *R* software (V.3.6.3) [21], and the fold change (FC) between the REG treatment group and the control group was computed to determine the DEGs. The screening thresholds for DEGs are as follows: (I) |log₂FC| > 1 and (II) *P*.adj < 0.05.The visualization results of the DEGs were presented in the form of volcano plots, heat maps, and Venn plots. The volcano plots and Venn plots analyzed all DEGs; however, due to the large number of genes, the heat maps analyzed the DEGs of the top 40 to make the results clearer and increase the legibility of the results.

RETRACTED

### 2.3. Gene Ontology (GO) Enrichment Analysis

GO enrichment analysis includes biological process (BP), cell composition (CC), and molecular function (MF) to supply functional information about DEGs in cardiomyocytes treated by REG compared with normal cardiomyocytes in the control group [22]. The clusterProfiler package (V.3.14.3) in *R* software (V.3.6.3) [23] was employed to perform GO analysis for DEGs; subsequently, for gene ID conversion, the http://org.Hs.eg.db package (V3.10.0) was downloaded from Bioconductor (https://bioconductor.org) [24]. GOplot package (V1.0.2) was used to calculate *z*-score, and the selected species for screening was Homo sapiens [25].

### 2.4. Kyoto Encyclopedia of Genes and Genomes (KEGG) Enrichment Analysis

KEGG enrichment analysis determines functional meanings and the route of the gene cluster of differential expression genes [26]. In order to make the data more intuitive and rigorous, we analyzed the DEGs' KEGG pathway enrichment using the DAVID database (DAVID version 6.8; https://david.ncifcrf.gov) and then visualized the results.

### 2.5. Gene Set Enrichment Analysis (GSEA)

The GSEA was utilized to examine and explain variations in the coordinate pathway levels of DEGs in REG-treated and normal cardiomyocytes [27]. First, we downloaded the GSEA software from http://software. http://broadinstitute.org/gsea/index.jsp. Then, the reference datasets were c2.cp.v7.2.symbols.gmt, which were retrieved from the Molecular Signatures Database (https://www.gsea-msigdb.org/). Subsequently, the clusterProfiler package (V.3.14.3) and ggpolt2 package (V.3.3.3) in *R* were utilized to perform GSEA analysis and visualize [23, 28]. The significant enrichment of GSEA analysis was established by the threshold values (FDR < 0.25 and *P*.adj < 0.05).

### 2.6. Cell Culture

AC16 human cardiomyocyte cell line was purchased from American Type Culture Collection (ATCC, Rockville, MD). Under conditions of CO_2_ incubators maintaining atmospheric oxygen levels and 5% CO_2_, cardiomyocyte cells were cultured using Dulbecco's modified Eagle's medium (DMEM, Gibco, 11965092, USA) with 10% fetal bovine serum (FBS, Gibco, 16140071, USA). Cells were passed regularly and subcultured to 80% confluence before the cell experiment. For 12 h prior to each experiment, the cell medium was supplemented with 0.5% FBS. A concentration of 1 *μ*M of regorafenib (HY-10331, New Jersey, USA) was then applied to the plates for 48 hours. Regorafenib was melted in dimethyl sulfoxide (DMSO, Biosharp, BS087, China), and DMSO was used as a control at a concentration of 0.1 nM.

RETRACTED

### 2.7. Real Time-qPCR

It was decided to utilize only total RNA that had been extracted from cells and mice tissues by following the manufacturer's procedure and then synthesizing it using the Transcriptor First Strand cDNA Synthesis Kit (Roche, 04896866001, Germany) and TRIzol Reagent (15596026, USA). Bio-Rad CFX96 Touch Real-Time PCR Detection System (Bio-Rad) and SYBR Green I Master Mix were used for RT-PCR analysis of RNA (Roche, 4707516001, Germany). Automated threshold cycles (Ct) were created and standardized to the GAPDH reference gene. 2^-*ΔΔ*Ct^ values are used to represent the data. All details of the PCR primer sequences are presented in Supplemental Table 1.

### 2.8. Development of Receiver Operating Characteristic (ROC) Curves

The ROC analysis was used to test the sensitivity and specificity of screened DEFRGs. The pROC package and the ggplot2 package in the *R* software are used with data analysis and visualization, respectively [29]. The area under curve (AUC) of the receiver operating characteristic (ROC) is between 0.5 and 1, with a value near 1 indicating excellent prediction capacity and a value of 0.5 suggesting no predictive power.

### 2.9. Statistics

The results are reported as the mean ± standard error of the mean (SD) of at least three separate experiments. Descriptive data and figures were prepared using GraphPad Prism (Version 8.0.2, GraphPad Software, La Jolla, CA, USA). Unpaired Student's *t*-tests were performed to compare the means of two groups, and *F*-tests for equality of variance were used for all *t*-tests to compare variances. *P* values of <0.05 were defined as statistically significant.

## 3. Results

### 3.1. Identification of Differentially Expressed Genes

To obtain DEGs that may cause cardiotoxicity with the anticancer drug REG, we, respectively, performed differential expression analysis of four groups of adult heart-derived primary cardiomyocytes from GSE146096 dataset using the DESeq2 *R* package [21]. Then, through the processing of the data, we get the volcano plots and heat maps of each set of difference expression analysis separately (Figure 2). After using |log₂FC| > 1 and *P*.adj < 0.05 as the cutoff value of screening, a total of 747 DEGs in 6 control groups and 2 REG treatment groups in A line were screened, of which were 246 genes highly expressed (log₂FC > 1) in the REG groups and 501 genes highly expressed (log₂FC < −1) in the normal groups (Figures 2(a) and 2(e)). Meanwhile, in B line, a total of 1127 DEGs were screened, with 545 genes expressing highly in the REG groups and 582 genes expressing highly in the normal groups (Figures 2(b) and 2(f)). A total of 773 DEGs in 6 control groups and 3 REG treatment groups in D line were screened, of which were 442 genes with expressing highly in the REG groups and 331 genes with expressing highly in the normal groups (Figures 2(c) and 2(g)), and a total of 969 DEGs in 11 control groups and 4 REG treatment groups in E line were screened, of which were 468 genes with expressing highly in the REG groups and 501 genes with expressing highly in the normal groups (Figures 2(d) and 2(h)). The top five upregulated and downregulated genes with high significant in each group are labeled separately in the plot. The results obtained by the four groups of DEGs intersected each other, and the results obtained by the four groups of upregulation genes and downregulation genes were shown in Figures 2(i)–2(k).

RETRACTED

### 3.2. GO Functional Enrichment Analysis

Based on *R* software, we executed the GO functional enrichment analysis to gain biological process (BP), cellular component (CC), and molecular function (MF) of DEGs of REG. The results for each line are shown in Figure 3. After a comprehensive assessment of *z*-score and the adjust *P* value, differentially expressed cardiotoxicity genes induced by REG in A line were significantly enriched in the muscle system process, extracellular matrix organization, collagen-containing extracellular matrix, cell-substrate junction, and extracellular matrix structural constituent (Figure 3(a)). Meanwhile, according to the same method, the DEGs in B line are significantly enriched in the muscle system process, muscle tissue development, stress fiber, contractile actin filament bundle and growth factor binding (Figure 3(b)); the DEGs in D line are significantly enriched in the regulation of binding, focal adhesion, cell-substrate adheres junction, cell-substrate junction, and actin binding (Figure 3(c)); and the DEGs in E line are mainly enriched in the regulation of smooth muscle cell proliferation, smooth muscle cell proliferation, transcription corepressor activity, and extracellular matrix component (Figure 3(d)).

### 3.3. KEGG Functional Enrichment Analysis

In this study, KEGG functional enrichment analysis results based on the DAVID database indicated that differentially expressed cardiotoxicity genes induced by REG were mainly enriched in focal adhesion, hypertrophic cardiomyopathy (HCM), PI3K-Akt signaling pathway, biosynthesis of amino acids, and dilated cardiomyopathy in A line (Figure 4(a)). In addition, the results showed that the DEGs in REG groups and normal groups in B line significantly enriched in TGF-beta, Rap1, focal adhesion, PI3K-Akt, and thyroid hormone signaling pathway (Figure 4(b)). And in D line, the DEGs were mainly enriched in glycolysis/gluconeogenesis, transcriptional misregulation in cancer, biosynthesis of amino acids, TGF-beta, and HIF-1 signaling pathway (Figure 4(c)). The DEGs in E line were significantly enriched in PI3K-Akt, MAPK, regulating pluripotency of stem cells, focal adhesion, and TGF-beta signaling pathway (Figure 4(d)).

RETRACTED

### 3.4. GSEA Enrichment

GSEA was performed to detect biological properties common to differentially expressed cardiotoxicity genes, using each line of DEGs as raw data. After GSEA enrichment by the A line differential gene set, we found that the selected gene set presented as low expression in the pathway NABA_MATRISOME (NES = −1.942, FDR = 0.110) and pathway REACTOME_MUSCLE_CONTRACTION (NES = −1.981, FDR = 0.110), the main function of the former being ensemble of genes encodes extracellular matrix and extracellular matrix-associated proteins, and the latter is related to muscle contraction (Figure 5(a)). Similarly, after our GSEA analysis of B line, we found that the differential genes in B line showed a low expression trend in both pathway NABA_MATRISOME (NES = −1.993, FDR = 0.058) and pathway REACTOME_ION_CHANNEL_TRANSPORT (NES = −2.182, FDR = 0.058) associated with ion channel transport (Figure 5(b)). However, the GSEA results in the D line showed that gene sets were highly expressed PID_ATF2_PATHWAY (NES = 2.222, FDR = 0.040) related to ATF-2 transcription factor network and low expression in KEGG_OXIDATIVE_PHOSPHORYLATION (NES = −2.336, FDR = 0.040) which participates in oxidative phosphorylation (Figure 5(c)). In E line, gene sets that encode extracellular matrix glycoproteins, collagens, and proteoglycans are expressed at low levels in the NABA_CORE_MATRISOME (NES = −2.497, FDR = 0.051), which is composed of an ensemble of genes that encodes the extracellular matrix glycoproteins, collagens, and proteoglycans and highly expressed in the PID_ATF2_PATHWAY (NES = 2.212, FDR = 0.051) (Figure 5(d)).

### 3.5. Validation and Functional Analysis of DEFRGs

After the four lines of A, B, D, and E differentially expressed cardiotoxicity genes were intersection, 122 common DEGs were obtained and then intersected with 259 ferroptosis-related genes collected from the FerrDb database, and 7 differentially expressed ferroptosis-related genes (DEFRGs) were obtained, including NADPH oxidase 4 (NOX4), DNA damage inducible transcript 4 (DDIT4), growth differentiation factor 15 (GDF15), solute carrier family 3 member 2 (SLC3A2), metallothionein 1G (MT1G), activating transcription factor 3 (ATF3), and perilipin 2 (PLIN2) (Table 1). Subsequently, in order to verify the above 7 DEGs, real time-qPCR and statistical analysis were performed on cultured cells, the specific results were shown in Figure 6, and ATF3 (*P* < 0.05), MT1G (*P* < 0.001), and PLIN2 (*P* < 0.01) were the prominent and upregulated genes, whereas DDIT4 (*P* < 0.05) was the notable and downregulated gene.

RETRACTED

Moreover, in order to further verify whether the above four DEFRGs can be used as target genes to predict REG-induced cardiotoxicity, we used ROC analysis to examine the sensitivity and specificity of DEFRGs, and the results showed that the upregulated genes ATF3 (AUC = 0.982, CI = 0.944 − 1.000), MT1G (AUC = 0.844, CI = 0.691 − 0.996), PLIN2 (AUC = 0.992, CI = 0.975 − 1.000), and downregulated genes DDIT4 (AUC = 0.945, CI = 0.875 − 1.000) all had high accuracy (Figures 7(a) and 7(b)). Based on the above results, the four DEFRGs (ATF3, MT1G, PLIN2, and DDIT4) all have sufficient confidence to prove that they are the key genes of REG-induced cardiotoxicity through the ferroptosis pathway. To be more crucial, this result provides new insights into the cardiotoxicity induced by REG that targets above four gene therapy.

## 4. Discussion

Earlier researches have confirmed that anticancer drugs play a pivotal role in ferroptosis-related cardiotoxicity [19] and have identified the possibility of prevention of cardiomyopathy by targeting ferroptosis [30].

Sorafenib is chemically similar to regorafenib [31], and sorafenib as a cystine-glutamate antiporter inhibitor can induce ferroptosis in cells by depleting cellular GSH [20]. By comparing 80 sorafenib-induced cardiotoxicity DEGs and 122 regorafenib-induced DEGs, we found that a total of 21 genes involved in inducing cardiotoxicity were found, including ATF3, metallothioneins (MTs), SLC3A2, GDF15, and PLIN2, which coincided with our findings, suggesting that regorafenib is the same as sorafenib and may induce cardiotoxicity through similar mechanisms. Furthermore, many studies have also shown that ferroptosis is indeed one of the potential mechanisms for inducing cardiotoxicity, such as Fang et al. demonstrating that ferroptosis, rather than other known forms of regulating cell death, plays a key role in doxorubicin-induced cardiotoxicity [30].

In this study, we first used the dataset of four adult human cardiomyocytes treated by REG as an entry point to seek correlation between the dataset after differential expression analysis and the ferroptosis genes, and finally, the four DEGs (ATF3, MT1G, PLIN2, and DDIT4) proved to be reliable prognostic biomarkers and future therapeutic targets for REG-induced cardiotoxicity. Based on this context, our study has some strengths over previous studies. First of all, we think that our biggest advantage is that we used four sets of experimental data in the same dataset to analyze the differences and then take the intersection, which not only overcame the shortcomings of the samples to a certain extent but also improved the accuracy of selecting the difference genes while taking the same truncation values. Secondly, we used a corrected *P* value to perform multiple hypothesis tests rather than the original *P* value to better control the false positive rate. Thirdly, we selected NOX4, DDIT4, GDF15, SLC3A2, MT1G, ATF3, and PLIN2 to verify their expression in REG-induced cardiotoxicity with real time-qPCR. The advantage is that it has a wider quantitative linear range than ordinary PCR, and the results showed that three DEGs (ATF3, MTIG, PLIN2) were upregulated and one DEG (DDIT4) was downregulated. However, mRNA levels of the other three DEGs (GDF15, NOX4, SLC3A2) were not significantly changed as we predicted. Finally, ROC models were established for the four DEGs (ATF3, MT1G, PLIN2 and DIDI4) that were validated, further validating the correlation with cardiotoxicity. These results advance our knowledge of the processes behind the cardiotoxicity produced by REG-related ferroptosis.

RETRACTED

REG involved in our study has been authorized by the FDA for the therapy of CRC, GIST, and HCC through targeting tumor cell growth and vasculature formation by potently inhibiting RTK VEGFR1, 2, and 3, TIE2, and PDGFR-b [32]. In addition, REG could inhibit colony-stimulating factor-1 receptor (CSF-1R) to disrupt tumor immunity [33]. Many clinical studies have reported that REG has considerable cardiovascular toxicity, one of which showed that hypertension and ischemia were the most significant cardiovascular events (the incidence was 36.8% and 8.6%, respectively) [34]. In our study, we for the first time screened out seven genes associated with cardiotoxicity and ferroptosis under the condition of REG treatment, which may guide clinical practice and further avoid REG-induced cardiovascular events by intervening these genes.

In the present study, we focused on exploring potential pathways for REG-induced cardiotoxicity, with the aim of understanding the effects of REG on molecular biology and the microenvironment in the therapeutic context to further identify potential pathways for prognosis and targeted therapy. We used multiple biological analysis methods to reveal that the anticancer drug REG altered the expression of ferroptosis genes for the first time. Experimental results from GO and KEGG analysis showed that the mechanism by which REG induces cardiotoxicity associated with ferroptosis may be regulated by PI3K-Akt signaling pathway, TGF-beta signaling pathway, and MAPK signaling pathways. Studies have shown that benazepril hydrochloride prevents the anticancer drug doxorubicin-induced cardiotoxicity by modulating the PI3K-Akt pathway, and studies demonstrated that activating the PI3K-Akt pathway can be used as a promising cardioprotective strategy; although, we first proposed the correlation between REG-induced cardiotoxicity and the PI3K-Akt pathway, but the specific mechanism of action is not yet clear [35, 36]. Happily, the correlation between TGF-beta signaling pathways and MAPK signaling pathways and cardiotoxicity is unquestionable, meaning that TGF-beta signaling pathways and MAPK signaling pathways also have the potential to serve as potential pathways for determining prognosis and treating REG-induced cardiotoxicity [37, 38]. According to GSEA analysis, the screened DEGs in A line were lowly expressed in muscle contraction, DEGs in B Line were lowly expressed in ion channel transport, and ensemble of genes encoding extracellular matrix-associated proteins and extracellular matrix was low expression in both A and B. The ATF-2 transcription factor network is highly expressive in both D and E, the oxidative phosphorylation pathway is low in D, and the encodes ensemble of genes core extracellular matrix are low in E line. Our findings provide information for the progress of REG-induced cardiotoxicity in identifying differently expressed genes and biological pathways.

RETRACTED

ATF3, a member of the ATF/cAMP response element-binding (CREB) protein family [39], functions as a stress-induced transcription factor. Previous studies have shown that at the time of cardiac stress and cardiotoxicity (e.g., heart failure, cardiac hypertrophy, dysfunction, and fibrosis), low-expression ATF3 is typically highly elevated [40, 41]. In addition, ATF3 promoted ferroptosis induced by erastin [42]. Notably, ATF3 has been shown to increase the sensitivity of gastric cancer cells to cisplatin by promoting ferroptosis by inhibiting Nrf2/Keap1/xCT signaling [39], but the role of ATF3 in inducing cardiotoxicity through ferroptosis is still unclear. Our findings suggest that REG may upregulate the expression of ATF3 by promoting ferroptosis and eventually induce cardiotoxicity. Thus, we confirmed the association of ATF3 and cardiotoxicity in our study, pointing to a possible therapeutic target for cardiotoxicity caused by REG-related ferroptosis.

MTs are a class of metal proteins with a low molecular weight and a high cysteine content that are significantly activated in response to a variety of stimuli, including metals, cytokines, and free radicals [43]. MT1G, the number of the MTs family, inhibits carcinogenic effects, represses metastasis, and promotes cell differentiation [44–46]. One study suggested that the interaction of low-expression MT1G with p53 inhibited proliferation and enhanced apoptosis of HCC cells [47]. However, in the treatment of patients with advanced HCC, tolerance to targeted drugs is an inevitable reality, studies have shown that inhibition of MT1G expression could enhance sorafenib sensitivity [43]. In our study, we found enhanced MT1G expression of REG-treated cardiomyocytes, suggesting that inhibition of MT1G may reduce the incidence of REG-induced cardiotoxicity through ferroptosis, but currently, we have no evidence of the MT1G expression in reducing REG tolerance.

Lipid homeostasis in cardiomyocytes relies on a critical balance between peripheral fatty acid uptake and mitochondrial *β*-oxidative depletion [48]. PLIN2 from the PLIN family is characterized by lipid droplet (LD) proteins in adipocytes, which is involved in lipid metabolism and transport, cytoskeletal organization, and intracellular transport and signal transduction; thus, it is implicated in the onset and progression of numerous malignancies, including kidney cell carcinoma and mammary carcinoma [49]. Furthermore, overexpressed PLIN2 had a high significance (*P* < 0.01) in our study, and we reasonably presumed that REG may induce the upregulation of its expression and promote cellular programmed ferroptosis, eventually leading to cardiotoxic effects. This is the study which indicates that the upregulation of the PLIN2 expression may lead to cardiotoxicity [48].

DDIT4 is induced under a diversity of stress conditions, including oxidative stress, endoplasmic reticulum stress, hypoxia, and starvation. Du et al. found that downregulation of DDIT4 results in chemical sensitivity and proliferative suppression, indicating that the p53 and MAPK signaling pathways are activated, revealing that downregulation of DDIT4 suppresses gastric cancer tumor development [50]. However, in our cultured cells treated with REG, downregulation of the DDIT4 expression may indicate the onset of cardiotoxicity. Additionally, baicalein upregulated DDIT4 and inhibited the proliferation of platinum-resistant cancer cells, showing that regulating DDIT4 may have good prospects in the field of chemotherapy.

Our findings corroborated that despite enhanced mRNA expression levels in three genes (NOX4, SLC3A2, and GDF15), there was no statistically significance compared to the control groups. NOX4 inhibits human mitochondrial respiration and ATP production, thereby impairing mitochondrial metabolism, thereby promoting oxidative stress and ultimately leading to cellular ferroptosis. SLC3A2 has a function in tumor development and management of oxidative stress by modulating amino acid transport mechanisms [51]. Cardiomyocyte-derived endocrine hormone GDF15 governs body development with locally cardioprotective effects, and the GDF15 expression is substantially elevated in cardiomyocytes after myocardial infarction and within hours after myocardial infarction [52]. At the same time, experimental evidence supports GDF15 as a prognostic and therapeutic target for several cardiovascular and metabolic disorders [53].

RETRACTED

Of course, like most bioinformatics network analysis studies of human diseases, this study has certain drawbacks. First, in the selection of experimental groups, we selected only one data set resulting in a relatively small number of cardiac tissue samples; second, this study lacked in vitro experiments because we have difficulties in obtaining individual-specific clinical data from public datasets, which does reduce the reliability of the outcomes to some extent. Additionally, it is yet unknown whether genes associated with ferroptosis are expressed differently in cardiotoxicity and play alternative regulatory functions. Nonetheless, NOX4, SLC3A2, and GDF15 expression upregulation was not statistically significant and inconsistent with our analysis, possibly considering the number of REG and control groups used for real time-qPCR confirmation, and additional investigation is required to add the number of REG and control groups, as well as the total quantity of data in each group, to be utilized to verify these findings. What is more, although previous studies have confirmed that regorafenib can cause ferroptosis, and some anticancer drugs can induce cardiotoxicity through the ferroptosis pathway, there is no literature to confirm that regorafenib can induce cardiotoxicity through the mechanism of ferroptosis; so, we will further verify the role and mechanism of regorafenib in ferroptosis later.

## 5. Conclusions

In this study, based on bioinformatics analysis, we revealed the relationship between the cardiotoxic effects induced by the anticancer drug regorafenib and ferroptosis and validated target genes associated with cardiotoxicity induced by regorafenib. After identifying 7 expressed genes in GES146096 using 4 sets of data with comprehensive bioinformatics analysis, we further demonstrated that three upregulated genes (ATF3, MT1G, PLIN2) and one downregulated gene (DDIT4) may play a key role in REG-induced cardiotoxicity. As a result, our results may serve as a foundation for further research into the mechanism of REG-induced cardiotoxicity, as well as clinical preventive and therapeutic targets.

RETRACTED

## Figures and Tables

**Figure 1:** Flow diagram of data collection and analysis in this study.

**Figure 2:** Verification of differentially expressed genes (DEGs) of anticancer drug regorafenib. (a) Volcano plot for DEGs in A line. (b) Volcano plot for DEGs in B line. (c) Volcano plot DEGs in D line. (d) Volcano plot for DEGs in E line. (e) Heat map for DEGs in A line. (f) Heat map for DEGs in B line. (g) Heat map for DEGs in D line. (h) Heat map for DEGs in E line. DEGs in control groups and treatment groups were defined by the cutoff value (|log₂FC| > 1 and *P*.adj < 0.05), upregulated genes were in red, and downregulated genes were in blue. (i) Venn plot of upregulated and downregulated differential genes in A, B, D, and E lines. (j) Venn plot of upregulated differential genes in A, B, D, and E lines. (k) Venn plot of downregulated differential genes in A, B, D, and E lines.

**Figure 3:** Gene Ontology (GO) enrichment analysis of differentially expressed genes. (a) GO enrichment analysis for DEGs in A line. (b) GO enrichment analysis for DEGs in B line. (c) GO enrichment analysis for DEGs in D line. (d) GO enrichment analysis for DEGs in E line. BP: biological process; CC: cell composition; MF: molecular function. The abscissa represents GO gene IDs, the ordinate represents -log_10_ (*P*.adjust), and the color represents *z*-score.

**Figure 4:** Kyoto Encyclopedia of Genes and Genomes (KEGG) pathway enrichment of differentially expressed cardiotoxicity genes in REG groups and normal groups. (a) KEGG enrichment analysis for DEGs in A line. (b) KEGG enrichment analysis for DEGs in B line. (c) KEGG enrichment analysis for DEGs in D line. (d) KEGG enrichment analysis for DEGs in E line. The abscissa represents genes counts, the ordinate represents enrichment pathways, and the color represents -log_10_ (*P*.adjust).

**Figure 5:** Gene set enrichment analysis (GSEA) of differentially expressed cardiotoxicity genes in REG groups and normal groups. (a) GSEA enrichment for DEGs in A line. (b) GSEA enrichment for DEGs in B line. (c) GSEA enrichment for DEGs in D line. (d) GSEA enrichment for DEGs in E line.

**Figure 6:** Relative gene expression verification of seven expressed ferroptosis-related genes. The expression of NOX4 (a), DDIT4 (b), GDF15 (c), SLC3A2 (d), MT1G (e), ATF3 (f), and PLIN2 (g) was measured by real time-qPCR. ^∗^*P* < 0.05; ^∗∗^*P* < 0.01, ^∗∗∗^*P* < 0.001 vs. control group by Student's *t*-test.

RETRACTED

**Figure 7:** (a) ROC curve for upregulated genes (ATF3, MT1G, and PLIN2). (b) ROC curve for downregulated gene (DDIT4). The AUC ranges from 0.5 to 1.0, with near 1.0 indicating perfect predictive ability. The horizontal axis shows specificity (false positive rate), and vertical axis shows sensitivity (true positive rate).

**Table 1:** Summary of differentially expressed ferroptosis-related genes in cardiotoxicity induced by the anticancer drug regorafenib in lines A, B, D, and E.

Gene	Line A		Line B		Line D		Line E	
	Log_2_FC	*P*.adj	Log_2_FC	*P*.adj	Log_2_FC	*P*.adj	Log_2_FC	*P*.adj
NOX4	-1.28728	0.0026744	-1.8955291	2.47*E*-10	-1.612354	0.0002549	-1.646528	4.36*E*-05
DDIT4	-1.10465	0.0286193	-1.6882671	1.04*E*-06	-1.205564	9.50*E*-11	-1.074215	0.001506141
GDF15	1.3054065	0.0002622	2.39358373	4.40*E*-20	2.5868351	1.46*E*-17	2.768344	2.79*E*-26
SLC3A2	1.677388	2.93*E*-05	2.91411253	1.32*E*-36	2.4279102	8.89*E*-06	3.524854	4.99*E*-72
MT1G	2.8172485	0.0286193	2.71673009	2.92*E*-09	2.6578518	0.0003305	1.73884	0.002175718
ATF3	3.0720072	2.01*E*-15	3.82781296	2.45*E*-28	2.2034991	6.38*E*-05	3.788277	8.23*E*-23
PLIN2	3.2399218	3.24*E*-32	3.48984679	2.01*E*-114	2.7328507	3.70*E*-05	3.000006	5.40*E*-38

## Data Availability

Publicly available datasets were analyzed in this study. The mRNA expression profiles were obtained from the GEO databases (https://www.ncbi.nlm.nih.gov/gds/), namely, GSE146096.

## Supplementary Materials

Supplementary 1 Supplemental Table 1: the primer sequences for RT-qPCR.

Supplementary 2 Supplemental Table 2: gene sample in GSE146096.
